The article "A Hybrid Matching Network for Fault Diagnosis under Different Working Conditions with Limited Data" was published in 2022. Journal: Comput Intell Neurosci.

# A Hybrid Matching Network for Fault Diagnosis under Different Working Conditions with Limited Data

**DOI:** 10.1155/2022/3024590

**Published:** 2022-07-01

**Authors:** Qiuchen He, Shaobo Li, Chuanjiang Li, Junxing Zhang, Ansi Zhang, Peng Zhou

**Affiliations:** ^1^School of Mechanical Engineering, Guizhou University, Guiyang 550025, China; ^2^State Key Laboratory of Public Big Data, Guizhou University, Guiyang 550025, China

## Abstract

Intelligent fault diagnosis methods based on deep learning have achieved much progress in recent years. However, there are two major factors causing serious degradation of the performance of these algorithms in real industrial applications, i.e., limited labeled training data and complex working conditions. To solve these problems, this study proposed a domain generalization-based hybrid matching network utilizing a matching network to diagnose the faults using features encoded by an autoencoder. The main idea was to regularize the feature extractor of the network with an autoencoder in order to reduce the risk of overfitting with limited training samples. In addition, a training strategy using dropout with random changing rates on inputs was implemented to enhance the model's generalization on unseen domains. The proposed method was validated on two different datasets containing artificial and real faults. The results showed that considerable performance was achieved by the proposed method under cross-domain tasks with limited training samples.

## 1. Introduction

Mechanical fault diagnosis plays a significant role in modern industry. Failures of machines are likely to result in an entire mechanical system collapse and production line downtime, as well as serious economic losses. Timely and accurate fault diagnosis has become an indispensable technology in modern industries to ensure the safe and reliable operation of mechanical systems [1–3].

Recently, deep learning has achieved considerable progress in computer vision [4, 5], speech and natural language processing [6], product defect detection [7], and road planning [8]. Expectedly, an increasing number of researchers have applied deep learning techniques to fault diagnosis and proposed intelligent fault diagnosis methods [9–16]. Hasan et al. [17] proposed an explainable AI-based model for bearings fault diagnosis. Sun et al. [18] developed a sparse autoencoder-based deep neural network for the fault diagnosis of induction motors, which realized accurate fault prediction. Li et al. [19] designed a two-layer Boltzmann machine to develop representations of the statistical parameters of wavelet packet transform for gearbox fault diagnosis. Ding et al. [20] applied a deep convolutional neural network (CNN) by using wavelet packet energy as the input to develop a bearing fault diagnosis system, with which they obtained reasonable fault detection performance. Zhang et al. [21] proposed a method based on deep learning that uses raw temporal signals as input, which achieved high accuracy under noisy conditions. Qiao et al. [22] built a dual-input model and achieved satisfactory antinoise and load adaptability based on a CNN and a long short-term memory neural network. The deep learning methods have discarded the traditional time-consuming and unreliable manual analysis, improving the efficiency of fault diagnosis [23–28] considerably.

The article "A Hybrid Matching Network for Fault Diagnosis under Different Working Conditions with Limited Data" was published in 2022. Journal: Comput Intell Neurosci.

Traditional deep learning methods can only achieve satisfactory results when the training set (source domain) and the test set (target domain) are in the same data distribution. In practical applications, however, due to the complexity of the working conditions of the mechanical system (load, motor speed, etc.), the training set and the testing set may have distinct distributions. The predictive performance of the deep learning models is greatly affected by these facts. To face this challenge, some transfer learning algorithms have been proposed to enhance the domain adaptability of the model. Zhang et al. [21] presented a novel algorithm based on deep learning to alleviate the degradation of the performance of intelligent fault diagnosis under noisy environments and different working loads. Yao et al. [29] designed a new model based on a Stacked Inverted Residual Convolution Neural Network to ensure the accuracy of the model in noisy environments. Hu et al. [30] proposed a data augmentation algorithm and presented a self-adaptive neural network to boost models' generalization ability. Lu and Yin [31] developed a transferable common feature space mining algorithm to extract the common features from multidomain data. Wu et al. [32] constructed a few-shot transfer learning method in variable conditions. Wei et al. [33] proposed multiple source domain adaptation methods to extract condition-invariant features for fault diagnosis.

Aside from the obstacle posed by cross-domain tasks, a limited training set is another challenge that restricts the practical application of deep learning fault diagnosis algorithms. Most of the deep learning methods require a large amount of labeled data for model training. However, in actual industrial application scenarios, collecting a huge amount of labeled data for every type of failure under each working condition poses a considerable challenge. To address this problem, some studies on mechanical fault diagnosis using limited labeled training data have been conducted. Wang et al. [34] presented an integrated fault prognosis and diagnosis method for the predictive maintenance of turbine bearings, which achieved reasonable performance under limited labeled data. Zhang et al. [35] applied the few-shot approach for fault diagnosis and designed an artificial neural network based on a Siamese network, achieving interesting results with limited data. Li et al. [36] designed a meta-learning fault diagnosis method (MLFD) framework using model-agnostic meta-learning, which has performed excellently under complex working conditions. Hang et al. [37] applied a two-step clustering algorithm and principal component analysis to improve classification performance in the case of unbalanced high-dimensional data. Li et al. [38] proposed a deep, balanced domain adaptation neural network, which achieved satisfactory results with limited labeled data. Duan et al. [39] proposed a novel data description support vector based on deep learning for unbalanced datasets.

The article "A Hybrid Matching Network for Fault Diagnosis under Different Working Conditions with Limited Data" was published in 2022. Journal: Comput Intell Neurosci.

As two important research directions of fault diagnosis, improving the model's generalization to new domains and performance under limited training samples has made good progress, respectively. However, the reports of studies combining these two directions are relatively rare to find. In this study, to achieve domain generalization under limited training samples, we proposed a hybrid matching network (HMN) designed by connecting a prototypical network to the bottleneck of an autoencoder for fault diagnosis to unseen domains with limited training samples.

Our model mainly consists of two parts: (1) the autoencoder regularizing the feature extractor of the model to reduce the risk of overfitting and (2) the matching network achieving the measurement of samples similarity. Besides, a novel strategy is implemented in the training process to improve the model's domain generalization.

The main contributions of this study can be summarized as follows:

1. A novel fault diagnosis method based on matching network and autoencoder, known as HMN, was proposed to face the cross-domain scenarios. In the tasks, the model was training on the source domain with limited data and testing on the unseen target domains without access to their distributions.
2. Dropout on the input layer with randomly changing rates was employed to improve the generalization ability of the model. Autoencoder was built to reduce the risks of model overfitting with limited training samples by regularizing the feature extractor of the network.
3. The well-designed algorithm can effectively cope with domain generalization (DG) fault diagnosis. Comprehensive experiments were designed and executed to prove the effectiveness of the proposed HMN with two bearing faults datasets containing artificial and real faults.

The article "A Hybrid Matching Network for Fault Diagnosis under Different Working Conditions with Limited Data" was published in 2022. Journal: Comput Intell Neurosci.

The rest of the paper is organized as follows. Autoencoder and prototypical networks are introduced in Section 2.  Section 3 describes the proposed method in detail.  Section 4 presents the experiments, results, and discussion. Finally, the conclusions are drawn in Section 5.

## 2. Autoencoder and Prototypical Network

### 2.1. Autoencoder

Autoencoder, an unsupervised learning method, uses a neural network to implement the representation learning task. Specifically, a neural network architecture designed to impose a bottleneck layer forces a compressed knowledge representation of the original input.

As shown in Figure 1, the autoencoder is mainly composed of two parts: an encoder and a decoder. The encoder function, which is denoted as *f*_*θ*_, enables the efficient computation of a feature vector *h*=*f*_*θ*_(*x*) from an input vector *x*. It is important to note that the dimensions of *h* are usually lower than the dimensions of *x*. Another parameterized function *g*_*θ*_, known as the decoder, maps the feature vector back to the input space, generating a reconstruction vector $\hat{x}=g_{\theta }\left(h\right)$.

A simplified autoencoder structure can be represented as a fully connected neural network with three layers, i.e., an input layer, a bottleneck layer, and an output layer. The parameter sets of the encoder and the decoder are trained simultaneously when performing the task of reconstructing the input as much as possible, i.e., minimizing reconstruction error $L\left(x,\hat{x}\right)$ which is usually described by MSE over training examples. For a training set {*x*^(*i*)^}_*i*=1_^*n*^, the reconstruction error of MSE is expressed as follows:

(1) $$\begin{array}{c} J_{\text{MES}}\left(\theta \right)=\frac{1}{n}\sum_{i=1}^{n}\left(\frac{1}{2}\left|x^{\left(i\right)}-{\hat{x}}^{\left(i\right)}\right|\right). \end{array}$$

If the input is normalized to [0,1], the cost function can be described as binary cross-entropy, which comes in the form below:

(2) $$\begin{array}{c} J_{\text{bc}}\left(\theta \right)=\frac{1}{\text{nm}}\sum_{i=1}^{n}\sum_{j=1}^{m}\left[x_{j}^{\left(i\right)}\log{\hat{x}}_{j}^{\left(i\right)}+\left(1-x_{j}^{\left(i\right)}\right)\log\left(1-{\hat{x}}_{j}^{\left(i\right)}\right)\right], \end{array}$$

where *x*_*j*_^(*i*)^ and ${\hat{x}}_{j}^{\left(i\right)}$ represent the *j* th element of *x*^(*i*)^ and ${\hat{x}}^{\left(i\right)}$, respectively, *n* and *m* represent the batch size and the dimension of *x*, respectively.

Using penalizing parameters based on reconstruction errors, the network can learn about the most important attributes of the input data and how to best reconstruct the input from the feature vector.

The article "A Hybrid Matching Network for Fault Diagnosis under Different Working Conditions with Limited Data" was published in 2022. Journal: Comput Intell Neurosci.

### 2.2. Prototypical Networks

Prototypical Networks [40] have been proposed for few-shot learning, which requires only a small amount of training data with limited information, as compared to traditional machine learning methods requiring a large amount of data to train a model for good results. As shown in Figure 2, the classification task can be achieved by comparing the distances with mean representations of each class in the metric space produced by Prototypical Networks.

Specific to a few-shot task, given a support set that has *M* labeled samples *S*={(*x*_1_, *y*_1_),…, (*x*_*M*_, *y*_*M*_)}, *x*_*i*_ ∈ *R*^*D*^ is a vector with *D*-dimension and *y*_*i*_ ∈ {1,…, *K*} is the label of each class, *S*_*k*_ describes the set labeled with *k*. A representation *c*_*k*_, or prototype, of each class is computed by meaning the support points belonging to class *k*:

(3) $$\begin{array}{c} c_{k}=\frac{1}{\left|S_{k}\right|}\sum_{\left(x_{i},y_{i}\right)\in S_{k}}f_{\theta }\left(x_{i}\right), \end{array}$$

where *f*_*θ*_ is an embedding function with learnable parameters *θ*. For a function computing distance *d*=*R*^*D*^ × *R*^*D*^⟶[0, +*∞*), distribution of a query point *x*_*q*_ over distances to all prototypes of each class in the metric space is computed by prototypical networks:

(4) $$\begin{array}{c} p_{\theta }\left(y=k|x_{q}\right)=\frac{\exp\left(-d\left(f_{\theta }\left(x_{q}\right),c_{k}\right)\right)}{\sum_{k^{\prime }}\exp\left(-d\left(f_{\theta }\left(x_{q}\right),c_{k^{\prime }}\right)\right)}. \end{array}$$

Train the network by minimizing *L*(*θ*)=−log*p*_*θ*_(*y*=*k|x*_*q*_), the loss of the *k* class.

## 3. Methods

The proposed HMN for fault diagnosis is described in detail in this section. As shown in Figure 3, our model has both one-input and two-output configurations. One of the outputs was the reconstruction of the input, and the other was the prediction of health conditions using a prototypical network. The details of the model are illustrated in Table 1.

### 3.1. Data Preprocessing

The proposed model used the short-time spectrogram as a 2D input. Firstly, as shown in Figure 4, the sliding window of 2048 points generated the samples. Secondly, STFT used a fixed-length nonzero window function to slide along the time axis, truncating the source signal into segments of equal length. Assuming that these segments are stable, Fourier transform can be used to obtain the local frequency spectra of the segments. And finally, these local frequency spectra were recombined along the time axis to obtain a 2D time-frequency graph. The formula is presented in equation (5) as below:

(5) $$\begin{array}{c} \text{STFT}=\int_{-\infty }^{+\infty }x\left(t\right)g\left(t-\tau \right)e^{-j\omega t}d\tau , \end{array}$$

where *x*(*t*) is the original timing signal and *g*(*t* − *τ*) is the window function applied as the center point at time *τ*. In this study, the Hann window was used. To speed up the convergence of the model, we converted 2D spectrogram into a grayscale image with a value between 0 and 1. This process can be expressed as follows:

(6) $$\begin{array}{c} X^{\prime }\left(\tau \text{,}\omega \right)=\frac{\left|X\left(\tau ,\omega \right)\right|-{\left|X\left(\tau ,\omega \right)\right|}_{\min}}{{\left|X\left(\tau ,\omega \right)\right|}_{\max}-{\left|X\left(\tau ,\omega \right)\right|}_{\min}}, \end{array}$$

where |*X*(*τ*, *ω*)| is the element magnitude, |*X*(*τ*, *ω*)|_min_ and |*X*(*τ*, *ω*)|_max_ represent the minimum and maximum magnitude, respectively. Finally, the normalized spectrogram *X*′(*τ*, *ω*) was compressed into 64×64 time-frequency graphs as the input of the model.

The article "A Hybrid Matching Network for Fault Diagnosis under Different Working Conditions with Limited Data" was published in 2022. Journal: Comput Intell Neurosci.

### 3.2. Random Dropout on Input

Dropout is a technique proposed in [41] to prevent the deep neural nets from overfitting. The key idea is to randomly deactivate the units along with their connections from the network with probability *p* during training, preventing units from coadapting too much. Applying dropout amounts to sampling a “thinned” network from the original one during training. During the testing phase, dropout is disabled, which can be seen as an average of the predictions of many “thinned” networks. The networks trained with dropout usually have much better generalization ability on supervised learning tasks.

The deactivated units affect all the ones in the network, including the layers with dropout. Dropout applied in the lower layers can also be seen as providing noisy inputs for the higher layers. It can be interpreted as a method of data augmentation by adding noise to its hidden layers.

Adding noise with a specific distribution was not enough. Inspired by [21], we randomly changed the dropout rate during the training to obtain noise with the uncertain feature. Specifically, in each batch of training, the dropout rate was a random value between 0.1 and 0.9. The visualization of the operation is illustrated in Figure 5.

(7) $$\begin{array}{c} p∼\text{Uniform}\left(0.1,0.9\right),\\ r_{i}∼\text{Bernoulli}\left(p\right),\\ \hat{x}=r_{i}*x. \end{array}$$

Here *∗* denotes an elementwise product. *r*_*i*_ is a vector whose elements follow independent Bernoulli random variable which has a probability *p*. *x* and $\hat{x}$ are the raw input and the interfered output of *x*.

The article "A Hybrid Matching Network for Fault Diagnosis under Different Working Conditions with Limited Data" was published in 2022. Journal: Comput Intell Neurosci.

The purpose of adding dropout to the input layer was to add masking noise to the input, making the model insensitive to disturbance and improving the domain generalization of the model.

### 3.3. Feature Extraction

To make full use of unlabelled information, an autoencoder was designed for feature extraction. In the encoding stage, the 2D time-frequency images first passed through a set of 2D convolutional layers. The 2D convolutional layers captured the localized features of the image well due to its translation invariance. To obtain more diverse features at the same feature level, the weights in the convolutional layer were designed as a series of 2D filters. Each filter convolves independently across the input feature map in the forward pass, obtaining the output of one of the convolution layer's channels. Generally, the computing of the convolutional layer *l* is expressed as follows:

(8) $$\begin{array}{c} Z_{c}^{l}=f^{l}\left(\sum_{i=1}^{c^{l-1}}W_{i,c}^{l}*Z_{i}^{l-1}+b_{c}^{l}\right), \end{array}$$

where *∗* operator denotes the convolution of the channel *i* of the feature matrix *Z*_*i*_^*l*−1^ and the kernel *W*_*i*,*c*_^*l*^, which produces the feature map *Z*_*c*_^*l*^ of the *c*^th^ channel of the layer *l*. *b*_*c*_^*l*^ is the bias of *c*^th^ channel in the layer *l*. The *f*^*l*^(·), a nonlinear activation function using RELU in this study is implemented on the final output of the convolution network.

The encoder and decoder were designed in a symmetrical form. To reconstruct the coding of the bottleneck layer to the same size as the input time-frequency image, a transposed convolution layer was used in the decoder to unsampled the feature map. Following [42], the encoder contained four convolution layers and two fully connected layers, while the decoder contained four transposed convolution layers and two fully connected layers.

### 3.4. Training of the Proposed Model

The two outputs of the model correspond to two different losses, including the reconstruction loss *L*_*r*_ computed by the autoencoder and the classification loss *L*_*c*_ computed by the prototype network. In the training process, *L*_*r*_ and *L*_*c*_ are minimized. The total loss in the model training can be described as follows:

(9) $$\begin{array}{c} L=L_{c}+\alpha L_{r}, \end{array}$$

where the hyperparameter *α* is the weight coefficient used to adjust the weights of different losses. In the training process, the network is optimized with an Adam optimizer which sets the learning rates for each parameter adaptively. The steps of the proposed training algorithm are listed in Algorithm 1.

## 4. Experiments, Results, and Discussion

### 4.1. Experiment Setup

#### 4.1.1. Experiment Description

To verify the validity of our method, experiments are carried out on two bearing datasets selected from the Case Western Reserve University (CWRU) bearing datasets [43] and Paderborn bearing dataset [44]. We assume the source domain contains limited labeled samples and set 6, 10, 15, 50, 100, 200, 300, 500, 600 training samples per class to test the performance of the proposed method. Fivefold cross-validation is applied to the experiments. The test platform uses an Ubuntu 18.04 + Python 3.6 + Pytorch with an Intel® CORE™ i7-9750H CPU and a Nvidia GTX 1080Ti GPU.

The article "A Hybrid Matching Network for Fault Diagnosis under Different Working Conditions with Limited Data" was published in 2022. Journal: Comput Intell Neurosci.

#### 4.1.2. Comparison Methods and Evaluation Metrics

To verify the advantages of the proposed model, as shown in Table 2, several popular models are compared, using three types of time series input methods (Siamese-based CNN [35], PSDAN [45], and WDCNN [46]) and three types of time-frequency input methods (SCNN, HCAE [42],s and DeIN [47]). The Siamese-based CNN was designed by [35]. PSADAN was an adversarial domain adaptation method. WDCNN, in which a wide convolution kernel was used in the front of the network, was proposed in [46]. DeIN was proposed in [47]. SCNN is a common CNN that follows a softmax at the end of the same structure with the encoder of HMN. The HCAE was proposed in [42]. The HMN model was proposed by our team.

All the models are trained in the source domain and tested in the unseen target domain. For the sake of fair comparison, the hyperparameters of models are carefully selected.

Several evaluation indicators are used to evaluate the performance of the proposed model in the following aspects: (1) accuracy, (2) precision, (3) *F*1 score (*F*1), and average *F*1 score (*αF*1). Precision, *F*1, and *αF* can be obtained using the following equations:

(10) $$\begin{array}{c} \text{Precision}=\frac{\text{TP}}{\text{TP}+\text{FP}},\\ F1=\frac{2\text{TP}}{2\text{TP}+\text{FN}+\text{FP}},\\ \alpha F1=\frac{\sum F1}{\text{Total}\_\text{classes}}, \end{array}$$

where TP, FP, and FN represent true positive, false positive, and false negative, respectively.

### 4.2. Case Study 1: CWRU Bearing Datasets

#### 4.2.1. Data Description

In the CWRU bearing datasets [43], the 12k drive end fault data were selected as the original experimental data. Four types of faults, i.e., normal, ball fault, inner race fault, and outer race fault, were found in these data, as shown in Table 3. Each fault type had three different subtypes, i.e., 0.007 inches, 0.014 inches, and 0.021 inches. Thus, there were altogether 10 different types of fault.

Signals of all fault types are shown in Figure 6. Each type of fault had three different loads, i.e., 1, 2, and 3 hp (motor speed of 1772, 1750, and 1730 RPM), as illustrated in Table 4. During data collection, each sample was collected from a vibration signal, as shown in Figure 7. Half of the signals were used to generate training data, and the remaining signals were used to generate the test set. As shown in Figure 4, the training samples were generated using 2048 points sliding window with 80 points overlapping steps. The test set samples passed through sliding windows in the same size, but the samples were generated without overlapping.

The article "A Hybrid Matching Network for Fault Diagnosis under Different Working Conditions with Limited Data" was published in 2022. Journal: Comput Intell Neurosci.

We set the data under different working conditions as experimental data. Datasets A, B, and C correspond to different working conditions with loads of 1, 2, and 3 hp, respectively. Each dataset contained 6000 training samples and 250 test samples.

#### 4.2.2. Results and Analysis

Figure 8 illustrates the accuracy of all methods of training with various amounts of samples. With outstanding performance, HMN is evidently superior to the other approaches. We can find that cross-domain task C to A is the most difficult, in which even with sufficient training samples, the accuracy of four compared methods does not reach 90%, but the proposed model still achieves satisfactory results.

The results of training with 6 samples per class were observed. The classification accuracies of the cross-domain tasks are shown in Table 5. The best performance was achieved using HMN among all the methods in all the scenarios. Specifically, HMN achieved an accuracy of 92.65% in C-A, which was 34.61%, 21.57%, 26.38%, 19.32%, 40.21%, and 27.09% higher than DeIN, Siamese Based CNN, WDCNN, SCNN, HCAE, and PSDAN, respectively.

In Tables 6 and 7, the precisions and *F*1 (*αF*1) of HMN and the other 6 methods in the cross-domain task C-A are compared, each training class containing 6 samples (the most difficult task). The results reveal that the suggested HMN outperformed all of the compared approaches. This evidenced that HMN can achieve more robust performance in cross-domain diagnostic tasks with limited training samples.

To further evaluate the effectiveness of the proposed method, we observed the effects of the autoencoder and random dropout in improving model's performance through the loss curve. Figures 9 and 10 show the loss curves in cross-domain task C-A with 6 training samples per class.

As shown in Figure 9, training losses containing reconstruction loss *L*_*r*_ and classification loss *L*_*c*_ are considered to originate from equation (9), with testing losses set to classification loss *L*_*c*_. According to equation (9), when *α* is set to 0, the autoencoder does not work. A greater *α* indicates a higher weight of autoencoder during the training process. As *α* increases from 0 to 0.2, the testing loss converges to a smaller value. The testing loss's convergence process is smoother when *α* equals to 0.5. This demonstrates how the autoencoder branch may prevent overfitting and improve the model's performance.

The article "A Hybrid Matching Network for Fault Diagnosis under Different Working Conditions with Limited Data" was published in 2022. Journal: Comput Intell Neurosci.

As shown in Figure 10, when the HMN does not employ random dropout on input, the convergence value of the testing loss is greater than 3; however, when random dropout is used, the convergence value of testing loss drops to less than 1, and the curve descends more smoothly. The effect of random dropout on input in improving the model's cross-domain generalization is demonstrated.

### 4.3. Case Study 2: Paderborn Dataset

#### 4.3.1. Data Description

As shown in Figure 11, the test rig [44] consists of five modules: (1) electric motor, (2) torque-measurement shaft, (3) rolling bearing test module, (4) flywheel, and (5) load motor. Bearings with different state types were installed in the test module to obtain experimental data. Fault types of bearings come from artificial and real damages.

In the basic setting of operating condition, the test platform ran at *n* = 1500 rpm with a load torque of *M* = 0.7 Nm and a radial force on the bearing of *F* = 1,000 N. Other settings were set up by changing the parameters one by one to *M* = 0.1 Nm and *F* = 400 N (named D, E, F, respectively, shown as Table 8.

The bearings with 32 different states were operated under different working conditions, including 14 states with natural damages from accelerated lifetime tests, 12 states with artificial damage, and 6 states with health data.

Each bearing under a load setting is measured with a vibration signal of about 4s at a 64 kHz sampling rate. In the experiment, datasets contained signals obtained from healthy bearings, artificially damaged bearings, and naturally damaged bearings. All bearings of different fault types were running under three different loads at a speed of 1500 rpm. The datasets filenames selected are shown in Table 9. The details of the datasets selected are listed in Table 10. Each dataset contains 1800 training samples and 120 test samples.

#### 4.3.2. Results and Analysis

By performing the same implementation, Figure 12 compares our method with the compared approaches in terms of the accuracy of different cross-domain tasks. The results show that our method outperformed the other six stat-of-the-art methods in all the scenarios.

Table 11 illustrates the cross-domain tasks accuracy of different methods with 6 training samples per class. The proposed method outperformed all comparative methods by 6.87%–41.26% on average. Tables 12 and 13 compare the methods in terms of precision, *F*1, and *αF*1 in the cross-domain task E-D with 6 training samples per class. The results also show that our method outplay the alternatives.

The article "A Hybrid Matching Network for Fault Diagnosis under Different Working Conditions with Limited Data" was published in 2022. Journal: Comput Intell Neurosci.

## 5. Conclusions

A novel HMN was proposed for cross-domain fault diagnosis with limited training samples. We improved the model's diagnostic performance in two ways: (1) a novel deep learning structure combining autoencoder and matching network was built, (2) a random dropout strategy adding random disturbance into the inputs during the training process was developed to enhance the model's domain generalization. In Section 4, we present the experimental results showing that the proposed method has better domain generalization ability with limited training samples compared with the state-of-the-art approaches.

However, the method proposed in this study still has some restrictions. For example, the method is limited to cross-domain tasks between different working conditions on the same device. However, cross-domain across multiple devices makes intelligent fault diagnosis algorithms more realistic. In addition, HMN can only perform classification tasks, limiting the model's potential to multitask. In future work, we will further optimize HMN and employ it in more complex cross-domain fault diagnosis scenarios and multitask learning.

## Figures and Tables

**Figure 1:** The typical architecture of a simple autoencoder.

**Figure 2:** Prototypical network. Prototypes *c*_*k*_ are the mean of the embedded support points. The embedded query points are classified via a softmax over distances to each prototype.

**Figure 3:** The architecture of the proposed model.

**Figure 4:** The vibration signal is sliced into samples containing 2048 points.

**Figure 5:** Input dropout:(a) without dropout, (b) with dropout.

**Figure 6:** Vibration signals corresponding to 10 states.

**Figure 7:** CWRU. Bearing fault diagnosis test rig.

**Figure 8:** The mean classification accuracy with the increasing number of training samples on CWRU. (a) Dataset A to dataset B. (b) Dataset A to dataset C. (c) Dataset B to dataset A. (d) Dataset B to dataset C. (e) Dataset C to dataset A. (f) Dataset C to dataset B.

**Figure 9:** Loss curves of the proposed model when *α* is set different values in cross-domain task dataset C to dataset A. (a) *α* = 0. (b) *α* = 0.2. (c) *α* = 0.5. (d) *α* = 0.8.

**Figure 10:** Loss curves: (a) training without random dropout; (b) training with random dropout.

**Figure 11:** Test rig of Paderborn bearing dataset.

**Figure 12:** The mean classification accuracy with the increasing number of training samples on the Paderborn dataset. (a) Dataset D to dataset E. (b) Dataset D to dataset F. (c) Dataset E to dataset D. (d) Dataset E to dataset F. (e) Dataset F to dataset D. (f) Dataset F to dataset E.

The article "A Hybrid Matching Network for Fault Diagnosis under Different Working Conditions with Limited Data" was published in 2022. Journal: Comput Intell Neurosci.

**Algorithm 1:** The proposed training algorithm.

**Table 1:** The details of the proposed networks.

Module	Layer	Layer type	Filter size/stride/channels (neurons)	Kernel number	Output size (Width*∗*Depth)
Shared encoder	1	Input	—	—	64*∗*64*∗*1
	2	Convolution	3*∗*3/2	16	32*∗*32*∗*16
	3	Convolution	3*∗*3/2	32	16*∗*16*∗*32
	4	Convolution	3*∗*3/2	32	8*∗*8*∗*32
	5	Convolution	3*∗*3/2	32	4*∗*4*∗*32
	6	Flatten	—	—	512
	7	Fully connected	64	—	64
	8	Fully connected	32	—	32
Decoder	9	Fully connected	64	—	64
	10	Fully connected	512	—	512
	11	Reshape	—	—	4*∗*4*∗*32
	12	Transposed convolution	3*∗*3/2	32	8*∗*8*∗*32
	13	Transposed convolution	3*∗*3/2	32	16*∗*16*∗*32
	14	Transposed convolution	3*∗*3/2	32	32*∗*32*∗*16
	15	Transposed convolution	3*∗*3/2	1	64*∗*64*∗*1
Matching	16	Prototypical loss	—	—	—

**Table 2:** Details of the comparison methods.

Input type	Method name	Implementation details
Time-based	Siamese based CNN	Details referred to [35]
	PSDAN	Implementation details referred to [45]
	WDCNN	Details referred to [46]

Time-frequency	SCNN	The encoder of HMN connecting softmax regression.
	HCAE	Implementation details referred to [42]
	DeIN	Details referred to [47]
	HMN (our)	As shown in Table 1

**Table 3:** Description of CWRU bearing datasets.

Fault location		None	Ball			Inner race			Outer race			Load
Fault Diameter(inch)		0	0.007	0.014	0.021	0.007	0.014	0.021	0.007	0.014	0.021	
Class labels		1	2	3	4	5	6	7	8	9	10	
Dataset A	Train	600	600	600	600	600	600	600	600	600	600	1
	Test	25	25	25	25	25	25	25	25	25	25	

Dataset B	Train	600	600	600	600	600	600	600	600	600	600	2
	Test	25	25	25	25	25	25	25	25	25	25	

Dataset C	Train	600	600	600	600	600	600	600	600	600	60 0	3
	Test	25	25	25	25	25	25	25	25	25	25	

**Table 4:** Three different working conditions.

Datasets	Load/HP	Rotational speed/rpm	Damage size/10^−3^in
A	1	1772	7, 14, 21
B	2	1750	7, 14, 21
C	3	1730	7, 14, 21

**Table 5:** Mean classification accuracy (%) with 6 training samples per class on CWRU.

Methods	A-B	A-C	B-A	B-C	C-A	C-B	Average
DeIN	90.14	53.76	62.33	72.17	58.04	62.76	66.53
Siamese based CNN	58.68	60.40	71.51	77.56	71.08	72.42	68.61
WDCNN	68.17	70.92	75.68	78.44	66.27	71.86	71.89
SCNN	89.14	69.15	85.15	80.44	73.33	82.56	79.96
HCAE	41.33	43.67	49.23	30.16	52.44	57.99	45.80
PSADAN	90.00	67.40	84.07	63.33	65.56	90.37	76.79
HMN (our)	**99.34**	**98.87**	**98.57**	**98.54**	**92.65**	**99.08**	**97.84**

**Table 6:** Precision (%) comparison for cross-domain task C-A with 6 training samples per training class on CWRU.

	Class 1	Class 2	Class 3	Class 4	Class 5	Class 6	Class 7	Class 8	Class 9	Class 10
DeIN	51.61	63.16	61.90	51.85	65.22	66.67	76.00	60.00	44.44	56.00
Siamese based CNN	75.00	81.48	80.77	67.86	72.73	50.00	65.38	73.91	70.00	80.00
WDCNN	65.38	60.00	64.00	56.52	69.57	77.78	66.67	69.23	66.67	68.42
SCNN	70.00	70.37	69.23	70.83	90.48	74.07	69.23	80.00	71.43	73.91
HCAE	55.56	55.26	40.00	44.00	40.00	52.17	57.69	66.67	54.84	66.67
PSADAN	56.52	84.21	55.56	50.00	61.11	76.92	75.00	72.73	66.67	72.41
HMN (our)	**88.46**	**92.59**	**87.50**	**92.31**	**100.00**	**89.29**	**96.00**	**88.46**	**100.00**	**95.65**

The article "A Hybrid Matching Network for Fault Diagnosis under Different Working Conditions with Limited Data" was published in 2022. Journal: Comput Intell Neurosci.

**Table 7:** *F*1 and *αF*1 (%) comparison with 6 training samples per class for cross-domain task C-A with 6 training samples per class on CWRU.

	Class 1	Class 2	Class 3	Class 4	Class 5	Class 6	Class 7	Class 8	Class 9	Class 10	*α*F1
DeIN	57.14	54.55	56.52	53.85	62.50	55.81	76.00	60.00	52.46	56.00	58.48
Siamese based CNN	66.67	84.62	82.35	71.70	68.09	52.83	66.67	70.83	76.36	71.11	71.12
WDCNN	66.67	65.45	64.00	54.17	66.67	80.77	65.31	70.59	69.23	59.09	66.19
SCNN	76.36	73.08	70.59	69.39	82.61	76.92	70.59	80.00	65.22	70.83	73.56
HCAE	46.51	66.67	43.64	44.00	35.56	50.00	58.82	55.81	60.71	60.87	52.26
PSADAN	54.17	72.73	57.69	61.54	51.16	78.43	58.54	68.09	72.73	77.78	65.28
HMN (our)	**90.20**	**96.15**	**85.71**	**94.12**	**93.62**	**94.34**	**96.00**	**90.20**	**95.83**	**91.67**	**92.78**

**Table 8:** Working conditions of rolling bearing on Paderborn.

Datasets	Rotational [rpm]	Load torque [Nm]	Radial force [N]	Name of setting
D	1500	0.7	1000	N15_M07_F10
E	1500	0.1	1000	N15_M01_F10
F	1500	0.7	400	N15_M07 _F04

**Table 9:** Data sets used for experiments.

Fault location	None	Out race	Inner race
File no.	K001	Artificial (KA01)	Artificial (KI01)
	K002	Real damages (KA04)	Real damages (KI14)

**Table 10:** Detail of datasets on Paderborn.

Dates sets	Splitting	None (class 1)	Inner race (class 2)	Out race (class 3)
D	Training	600	600	600
	Testing	40	40	40

E	Training	600	600	600
	Testing	40	40	40

F	Training	600	600	600
	Testing	40	40	40

**Table 11:** Mean classification accuracy (%) comparison with 6 samples per class on the Paderborn dataset.

Methods	D-E	D-F	E-D	E-F	F-D	F-E	Average
DeIN	66.57	70.47	66.41	61.57	42.37	43.21	58.43
Siamese based CNN	78.33	72.16	71.66	67.50	68.66	75.83	72.36
WDCNN	75.00	78.33	70.83	72.16	69.16	67.50	72.16
SCNN	67.83	69.03	56.82	64.27	58.34	57.63	62.32
HCAE	33.34	45.86	33.33	38.33	38.56	38.37	37.97
PSADAN	79.47	41.91	70.16	71.35	71.14	71.36	67.57
HMN (our)	**84.06**	**81.20**	**73.53**	**76.00**	**81.13**	**79.46**	**79.23**

**Table 12:** Precision (%) comparison for cross-domain task E-D with 6 training samples per class on the Paderborn dataset.

	Class 1	Class 2	Class 3
DeIN	62.00	69.23	70.97
Siamese based CNN	81.25	74.36	63.27
WDCNN	67.44	75.76	70.45
SCNN	60.00	56.82	56.10
HCAE	36.36	31.11	33.33
PSADAN	69.04	75.00	68.42
HMN (our)	**75.00**	**76.19**	**71.05**

The article "A Hybrid Matching Network for Fault Diagnosis under Different Working Conditions with Limited Data" was published in 2022. Journal: Comput Intell Neurosci.

**Table 13:** F1 and *α*F1 (%) comparison for cross-domain task E-D with 6 training samples per class on the Paderborn dataset.

	Class 1	Class 2	Class 3	*α*F1
DeIN	68.89	68.35	61.97	66.41
Siamese based CNN	72.22	73.42	69.66	71.77
WDCNN	69.88	68.49	**73.81**	70.73
SCNN	56.00	59.52	56.79	57.44
HCAE	32.88	32.94	34.15	33.32
PSADAN	70.73	75.00	66.67	70.80
HMN (our)	**75.00**	**78.05**	69.23	**74.09**

## Data Availability

The data used to support the findings of this study are available from the corresponding author upon request.
